# Perceptual-Cognitive Tasks Affect Landing Performance of Soccer Players at Different Levels of Fatigue

**DOI:** 10.1155/2022/4282648

**Published:** 2022-06-14

**Authors:** Yuanyuan Ren, Guodong Wang, Lei Zhang, Aming Lu, Cenyi Wang

**Affiliations:** Physical Education and Sport Science, Soochow University, China

## Abstract

**Background:**

There is a possible interaction between the underlying mechanisms of perceptual-cognitive tasks and motor control. For example, landing biomechanics changed during perceptual-cognitive tasks undertaken at different levels of fatigue of the athlete. Thus, this study explored the effect of perception-cognitive tasks interventions on male soccer players' landing mechanisms at different levels of fatigue.

**Methods:**

Perceptual-cognitive tasks during games were simulated using classic multiple object tracking (MOT) paradigms, and 15 male soccer players completed MOT tasks under nonfatigue (NF), moderate fatigue (MF), and severe fatigue (SF). Landing-associated indicators were collected and calculated using a Vicon and force measuring platform.

**Results:**

Level of fatigue and MOT task significantly affected hip and knee flexion angles, hip and knee extension moments, and vertical ground reaction force. Specifically, hip and knee flexion angles were significantly higher in MOT than non-MOT tasks at all levels of fatigue. In NF state, hip and knee extension moments were significantly smaller during MOT than non-MOT tasks. In SF state, the hip extension moment was larger during MOT than non-MOT tasks. In both MF and SF states, vertical ground reaction force was significantly higher in MOT than non-MOT tasks.

**Conclusion:**

Although soccer players landed cautiously when not fatigued, they were significantly less able to do this and handle challenging perceptual-cognitive task movements when fatigued. Thus, landing performance is affected by perceptual-cognitive task interference in fatigue conditions.

## 1. Introduction

As with visual attention features and dynamic tracking scenes, perceptual-cognitive expertise in interactive sports is highly relevant. A pertinent perceptual-cognitive task is multiple object tracking (MOT), which is the ability to divide attention and dynamically track multiple moving objects, such as in team sports when players need to concurrently focus on the position of the ball, teammate, and opponent [1]. MOT contributes largely to performance of voluntary movements that ensure success in team sports [1]. MOT mainly involves dynamic attention processing that utilizes perception-cognitive fields such as visual attention [1].

There is a possible interaction between mechanisms of perceptual-cognitive tasks (e.g., selective visual attention) and motor control—this has resulted in MOT tasks recently gaining extensive attention [2–4]. Indeed, the injury rate of soccer players was 14.4% higher in matches than routine training, and this difference was hypothesized to result from MOT tasks in soccer games [2]. More so, attention processing and neurocognitive abilities involved in MOT tasks are causative factors for impaired landing modes and high risks of injury [5]. From the U-shaped model theory, the relationship between cognition and postural control is a dual process, and individual postural control is related to cognitive task demands [6, 7]. During low cognitive task demand, individuals improved postural control by shifting their focus of attention away from highly automated activities. During high cognitive demands, two MOT tasks experienced intense resource competition, which negatively affected postural control ability [6, 7]. According to recent scientific studies, the body of knowledge on relationships between the functional state—a pertinent one is fatigue, which is a typical physiological and psychological phenomenon in continuous exercise—and cognitive performance of the human body during exercise has decreased with support for the hypothesis that exercise intensity produces linear changes in brain physiology and executive function [8–10]. Indeed, exercise-induced fatigue influenced landing movements and prolonged exercise dynamically influenced executive function [8, 9]. Moreover, exercise intensity and duration affected individual cognitive and executive functions [10]. Even more, different exercise intensities influenced cognitive and motor control changes during the acute exercise phase of subjects, because, when individual exercise intensity reached between 40% and 60% VO_2_max, the behavior accuracy of subjects was affected [11]. A dynamic-fatigue model explained this phenomenon: the executive function and movement performance of individuals during exercise changed from benefit to damage, and the duration of exercise was a key contributor to this [12]. Although previous studies have compared the effects of a single (motor only) and dual task (cognition and motor) on athletic performance [13–15], the effects of perceptual-cognitive task intervention on lower extremity landing patterns and risks of injury under different levels of fatigue remain unknown.

Therefore, this study was aimed at elucidating the impact of perceptual-cognitive tasks on landing performance and further investigated whether different levels of fatigue affected landing biomechanics in completing dual tasks (MOT and landing tasks). We hypothesized that perceptual-cognitive tasks affect landing performance: athletes perform better and are more able to maintain motor control and controllable landing mode when compared to when fatigued. Soccer players in the fatigued state had lower hip and flexion angles during the MOT task.

## 2. Methods

### 2.1. Participants

This study was approved by research ethics committee of the university(No. ECSU-2019000209). Fifteen college soccer male athletes—only male athletes were recruited as gender is one of the factors affecting landing biomechanics [16–18]—were enrolled in the study (height: 181.43 ± 7.36 cm, weight: 75.37 ± 10.67 kg, age: 20.07 ± 1.53 yr, and training years: 10.07 ± 2.98 yr). G-Power software was used to estimate the sample size which was a minimum of 12. Statistical significance was determined at an *α* level of 0.05, and thresholds for effective size and power of the statistical test (1-*β* err prop) were set at 0.25 and 0.95, respectively. Taking into account a possible sample loss rate of 10%, 15 people were enrolled, having met the following selection criteria: (1) athlete previously participated in provincial/large competitions and won a prize; (2) athlete had had no disease/injury in lower extremity joints in the past 6 months; and (3) athlete had not undertaken strenuous exercise within in the past 24 h preceding the test.

### 2.2. Experimental Setup

Landing tests were performed on a force platform (Kistler company, Switzerland), which detected ground reaction force. Vicon, consisting of 8 infrared cameras (Vicon, Inc., Oxford, United Kingdom) at a sampling rate of 100 Hz, was used to capture kinematic data. To define joint coordinate systems, a plug-in gait biomechanical model in Vicon was used, and markers were attached (Table 1). To reduce human errors, experimental data was collected by trained professionals.

### 2.3. Experimental Protocol

Participants warmed up by jogging at 4 km/h for 5-10 minutes on a treadmill. For the experiments on performance of perceptual-cognitive tasks, a 3D projector (Panasonic BX30, Panasonic Inc., Osaka, Japan) and screen were placed directly in front of the participants. The MOT task was given via bespoke programs written through Unity software (Unity Technologies, San Francisco, California, USA), which were projected on a 220 cm screen (Figure 1). The distance between the participant and screen was 130 cm (for both MOT and landing tasks) [19].

An MOT task was used that included eight identical spheres that interacted dynamically in a three-dimensional space—bounced off each other, broke the virtual three-dimensional volume boundary, and blocked each other. The task had four steps. First, eight randomly arranged identical spheres were presented on the screen. Second, the color of target spheres changed. Third, the color of all spheres reverted to the original color, and spheres then moved randomly on the screen at a uniform speed. Finally, participants pointed out the position target spheres (Figure 2). All subjects were asked to perform MOT task tracking test before the experiment, and the fastest tracking speed for the MOT task was recorded as initial speed. To ensure a similar MOT task load, the moving speeds of target spheres were adjusted to each participant's threshold and 30% of this speed was used for the test, to ensure that all participants can perform dual tasks (landing task and MOT task) [5, 19]. To reduce the learning effect, each participant was required to fully master the MOT task.

During experiments, participants were instructed to stand on 40 cm platforms with hands on hips and feet upright. Following the “start” signal, participants used dominant legs to step forward; then, they leaned forward and fell vertically from the steps, without initial speed, with grounding method and adopting “toe-heel” modes (Figure 3). Durations for landing and MOT tasks were equal with both tasks being completed simultaneously. The participants completed landing movements and MOT or non-MOT tasks synchronously. If the participants finished tasks sequentially, the run was not considered.

To determine levels of fatigue, the jump height (H) of the participants was calculated according to the formula *H* = 1.225T^2^ [20, 21], and the flight time (T) was measured by Vicon. The fatigue level was defined as the average decay rate of the vertical jump height plus the rating of perceived exertion (RPE) [22]. We divided fatigue into three levels: nonfatigue (NF); moderate fatigue (MF), whose decay in vertical jump height was 30% and RPE = 14 − 16; and severe fatigue (SF), whose decay in vertical jump height was 50% and RPE > 17. The fatigue induction method of “running + jumping” was selected because it is often experienced in soccer. In the fatigue intervention scheme, participants were required to perform six sets of 10 m shuttle runs at their maximum speed, quickly ran back to the force platform, and do five consecutive maximum jumps (Figure 4). The number of sets performed by each participant was determined by fatigue level.

### 2.4. Experimental Process

Participants completed landing movements while randomly doing MOT or non-MOT tasks in NF states. They were allowed to sufficiently rest between sets. Then, participants performed a fatigue intervention, in which they were not allowed to rest after it commenced. When participants reached targeted levels of fatigue (MF or SF), they immediately undertook landing tests with MOT or without MOT tasks, and they did approximately six drop landings (three MOT tasks and three non-MOT tasks) at each fatigue level. For example, when participants reached the MF level, they immediately performed both MOT or non-MOT tasks at random and synchronous landing actions and subsequently continued to complete the fatigue intervention program until they reached SF level. Immediately, they once again undertook both MOT and non-MOT tasks at random and synchronous landing actions. To minimize recuperation, avoid recovery, and maintain fatigue levels throughout the fatigued trials during landing tasks, participants performed additional five consecutive maximum vertical jumps between each landing undertaken with MOT or non-MOT task at each fatigue level.

### 2.5. Data Processing

The data was calculated by Visual 3D software via inverse dynamics method. Due to the high risk of injury at the time of first peak (the time corresponding to the first peak of the vertical ground reaction force curve) during the landing [23], we focus on this moment of landing change, with joint angle defined as 0° when the body is upright. At the time of first peak, an indicator of ground reaction force is vertical ground reaction force (VGRF). As different landing legs (dominant and nondominant legs) cause discrepancies in landing biomechanics [16, 24–26], we limited data to the dominant leg.

### 2.6. Statistical Analysis

Shapiro-Wilk tests and studentized residual method were used to determine normality and detect outliers, respectively. For normal data, sample means were tested using two-way repeated measures ANOVA to determine if they significantly differed. The study observed the main effect and interaction effects of different fatigue states (NF, MF, and SF) and MOT tasks (non-MOT task/MOT task) on biomechanical parameters. Subsequent multiple comparisons were performed by the least significant difference (LSD) method. Significance was set at *P* < 0.05.

## 3. Results

All data was normally distributed. There were significant effects of MOT task on the hip flexion angles (*P* = 0.001), knee flexion angles (*P* = 0.001), and knee valgus angles (*P* = 0.001). The hip flexion angles and knee flexion angles were significantly higher in MOT than non-MOT tasks, at all fatigue levels. The knee valgus angles were significantly higher in MOT than non-MOT tasks, only in NF and SF states (Figure 5).

There was a significant interactive effect of fatigue status and type of task on hip and knee extension moments (*P* = 0.012 and *P* = 0.030, respectively). Fatigue state and MOT task significantly affected on hip and knee extension moments. In NF state, the hip and knee extension moments were significantly lower in MOT task decreased than non-MOT task (*P* = 0.030). However, in SF state, the hip extension moment was higher in MOT than non-MOT tasks (Figure 6). Moreover, the hip extension moment was significantly higher in SF than NF (*P* = 0.001) under non-MOT task. Under MOT tasks, the knee extension moment was significantly higher in MF than NF (*P* = 0.012), and hip extension moment was significantly higher in SF than NF (*P* = 0.018).

VGRF was significantly higher in MOT than non-MOT task (*P* = 0.001) in both MF and SF states (Figure 7). However, VGRF had no significant differences in NF states.

## 4. Discussion

As expected, MOT task significantly affected biomechanics indicators of the lower extremity during landing such as the hip flexion angles, knee flexion angles, hip and knee extension moments, and VGRF. In NF state, the hip knee flexion angles were significantly higher in MOT than non-MOT tasks. Great hip and knee flexion angles, during landing, adjusted hip and knee extensor muscles for better absorption and reduction of impacts of ground reaction forces [27]. This indicates that soccer players might adopt a cautious landing strategy under MOT tasks. In contrast, soccer players seem to adopt a relatively rigid landing strategy in both MF and SF states of fatigue.

In MF and SF states, the hip and knee extension moments were higher in MOT than non-MOT tasks. Hip and knee extension moments were pivotal risk factors of noncontact ACL injuries [28, 29], which suggests that a deteriorative landing pattern may have occurred. This study further analyzed VGRF indicators and showed that in MF and SF states, larger VGRF was experienced in MOT than non-MOT tasks. According to previous studies, the increase of ground reaction force during landing might also be one of the factors causing the increase in joint moment and stiffness of the lower extremity [30]. VGRF is significantly correlated with vertical tibial peak and forward tibial shear forces when individuals land in the sagittal plane. The increase of VGRF caused a greater forward tibial shear force [31], demonstrating that high impact forces would be transmitted to the lower leg along the calcaneus and talus, and more loads would directly act on the bones and ligaments around the lower extremity joints [32]. Therefore, it appears that the landing performance is possibly affected by MOT task interference under fatigue, despite their desire to land in a protective manner, such as hip and knee extension moments and VGRF were individually impaired by MOT task interference at moderate to severe levels of fatigue. This result is similar to a previous study in which Mejane et al. [5] also confirmed that performing MOT tasks under fatigue induces adverse changes in lower extremity landing biomechanics. Although this high workload reduced physical output efficiency and also weakened behavior associated with the ideal judgment of perceptual-cognitive skills [23, 33], there seems to be a small magnitude of difference between groups. It suggests that the MOT task may not have greatly affected their landing mechanics. This may consider that soccer players were able to handle this cognitive task after prolonged dual-task training in games, and additional controlled studies are needed in the future to confirm this idea.

Our previous study has shown that in soccer players, postural stability and balance deteriorated during landing and MOT dual tasks [19]. The decrease in postural stability may also be the cause of reduced landing performance. This has been explained using a related theoretical model of capacity sharing [32]. Frontal lobe resources compete with each other between perceptual-cognitive tasks (MOT task) and motor-related demands (landing task), with participants prioritizing one task (MOT task) by reducing self-control task (landing), which impaired their postural control. Indeed, team sport athletes had to regularly extract and process information in their line of sight, and these specific cognitive functions (MOT tasks) deteriorated when exposed to higher stress levels (during games or competitions), which led to a decline in attention control ability [2]. This suggests that individual neuromuscular activity during an MOT task may not effectively control this challenging dual task. Furthermore, athletes at MF and SF states were less able to maintain favorable motor control, suggesting that the reason might be related to attention focus theory [34]. Repeated simple action execution allows individuals to process more peripheral sensory signals. In NF, the brain controls attention and muscle activity with relative ease, mainly through top-down attention strategies. For instance, people read when speaking, indicating that central motor commands automatically control most physical activities in daily life. The perception of movement and movement-related body sensations does not enter focus consciousness [35]. Thus, accordingly, subjects in NF state (manageable workload) effectively concentrated their attention, flexibly switching attention between the two tasks. While during exercise, the cumulative physical and cognitive demand is most often above the limit, and the execution efficiency becomes adversely affected [12]. In SF state (heavy workload), the attention of subjects was focused on the overwhelming physiological sensation, which dominated the focused consciousness and made them gradually lose their attention on their physical activities and motor control senses [36], thus causing some adverse changes in landing movements.

In addition, the recent research found that long-term MOT training has improved soccer players' athletic performance and decision-making ability [2]. Long-term MOT training positively affects motor stability and improves landing movement. It has been used for optokinetic simulation training, which possibly improved posture stability in dual tasks [2, 37]. Therefore, much more training-related research needs to be conducted in this field in specific populations for robust training recommendations.

There are still some limitations in this study. First, we did not use a parallel group for randomized control and did not randomize the fatigue state. Another limitation is that data on executive function was not collected, obscuring knowledge of the effect of the experimental design on frontal lobe resources during the MOT tasks. These issues should be considered and avoided in future research.

## 5. Conclusions

A cautious landing mode was adopted indicating athletes may be able to cope with this cognitive demand. However, fatigued soccer players possibly lack sufficient neuromuscular activity to control challenging movements during perceptual-cognitive tasks.

## Figures and Tables

**Figure 1:** Overview of the experimental setup.

**Figure 2:** MOT task experimental process.

**Figure 3:** Schematic diagrams of landing mode.

**Figure 4:** Schematic diagram of fatigue intervention scheme.

**Figure 5:** Changes of lower extremity joint angles. Note: ∗ means the indicators under MOT task are significantly different compared with no task, *P* < 0.05; # means the indicators in MF and SF are significantly different compared with NF, *P* < 0.05; *Δ* means the indicators in NF and SF are significantly different compared with MF, *P* < 0.05, the same as below.

**Figure 6:** Changes of lower extremity joint moment.

**Figure 7:** Changes of ground reaction force.

**Table 1:** Description of the paste position of the markers.

Position	Description
Bilateral anterior superior iliac spines	Anatomical position
Bilateral posterior superior iliac spines	Anatomical position
Bilateral proximal thigh	1/3 of the distance from hip to knee
Bilateral distal thigh	2/3 of the distance from hip to knee
Midlateral thigh	The middle of the lateral thigh from the hip to knee
Lateral condyles of both knees	Anatomical position
Bilateral proximal calf	1/3 of the distance from knee to ankle
Bilateral distal calf	2/3 of the distance from knee to ankle
Lateral middle of the calf	The middle of the lateral calf from knee to ankle
Bilateral lateral malleolus	Anatomical position
Bilateral calcaneus	Anatomical position
Bilateral second phalanges	Anatomical position

## Data Availability

The manuscript contains data.
